# Asymptomatic versus symptomatic solid pseudopapillary tumors of the pancreas: clinical and MDCT manifestations

**DOI:** 10.1186/s40644-019-0198-4

**Published:** 2019-03-07

**Authors:** Shudong Hu, Heng Zhang, Xian Wang, Zongqiong Sun, Yuxi Ge, Gen Yan, Changyong Zhao, Kemin Chen

**Affiliations:** 1 Department of Radiology, Affiliated Hospital, Jiangnan University, No. 200, Huihe Road, Wuxi, 214062 Jiangsu China; 2 Department of Radiology, Affiliated Renmin Hospital, Jiangsu University, No. 8, Dianli Road, Zhenjiang, 212002 Jiangsu China; 3 Department of General Surgery, Affiliated Hospital, Jiangnan University, No. 200, Huihe Road, Wuxi, 214062 Jiangsu China; 4 Department of Radiology, Ruijin Hospital, Shanghai Jiao tong University, School of Medicine, No. 197, Ruijin Er Road, Shanghai, 200025 China

**Keywords:** Incidental lesions, Solid pseudopapillary tumor, Pancreas, Computed tomography

## Abstract

**Background:**

To delineate the features of multi-detector computed tomography (MDCT) images and clinical characteristics of pancreatic solid pseudopapillary tumors (SPTs) of the pancreas in asymptomatic patients and compare these features and characteristics between asymptomatic and symptomatic patients.

**Methods:**

This work is a retrospective study approved by our institutional review board. MDCT images and clinical data of 109 patients with pathologically proven SPTs obtained from October 2008 to October 2016 were reviewed. Patients were categorized into two groups: asymptomatic patients and patients with symptomatic disease. Cases were reviewed to determine the reason for detection, intervention, shape, diameter, location, calcification, encapsulation, internal composition, CT attenuation, enhancement pattern, and tumor pathology. Clinical factors and imaging features were also compared between groups. Statistical analysis was performed using χ2 and t-tests.

**Results:**

Data from 49 asymptomatic and 60 symptomatic patients were collected. Asymptomatic SPTs were identified most frequently during routine health examination (18 patients, 36.7%), various screening purposes (12 patients, 24.5%), and traumatic injury (9 patients, 18.4%). Except for a smaller tumor size (5.8 cm in asymptomatic SPTs vs. 7.4 cm in symptomatic SPTs, *P* = 0.023), the clinical factors or imaging features of asymptomatic patients were very similar to those of symptomatic patients.

**Conclusions:**

The current research is the first single-center study to characterize SPTs in asymptomatic patients. Asymptomatic SPTs are gradually being identified with greater frequency. Although generally smaller in size than that in symptomatic patients, an asymptomatic pancreatic mass with the typical imaging features of SPT may be found, the treatment for which is similar to that for symptomatic patients. Evaluating asymptomatic SPTs requires further systematic and multi-center trials.

## Background

Solid pseudopapillary tumors (SPTs) of the pancreas used to be called Frantz tumors, solid cystic tumors, or solid pseudopapillary neoplasms. These tumors predominantly affect young female patients and usually have a favorable prognosis [1, 2].

The widespread use of cross-sectional imaging techniques, including multi-detector computed tomography (MDCT) and magnetic resonance imaging (MRI), has led to increased detection of cystic lesions of the pancreas in asymptomatic patients [3–6]. Approximately 15% of all patients undergoing abdominal MRI for other indications harbor unsuspected pancreatic cysts [7]. Asymptomatic cystic lesions of the pancreas are a rapidly increasing clinical entity, and pancreatic operations for asymptomatic patients are likely to become common, especially considering that a substantial proportion of these lesions may be malignant or of malignant potential [3, 5, 8, 9]. Once detected, the cysts can trigger significant anxiety for patients and their physicians [10, 11]. Immediate surveillance and evaluation and the resulting appropriate interventions can be invasive, expensive, and harmful. Information regarding asymptomatic cystic lesions of the pancreas is often sporadic, and previously published papers have mostly focused on serous cystadenomas, mucinous cystadenomas, mucinous cystadenocarcinomas, nonfunctional neuroendocrine tumors, and intraductal papillary mucinous neoplasms of the pancreas [3–5, 7, 10, 12]. To the best of our knowledge, comprehensive guidelines for the diagnosis and management of asymptomatic SPTs of the pancreas remain uncertain [13], In fact, only sporadic reports and guidelines represent the available literature on asymptomatic SPTs [10, 11]. Since a lack of prospective randomized trials exists in this field, no strong evidence is yet available today. The clinical and radiological characteristics of SPTs have yet to be fully clarified in asymptomatic patients; thus, asymptomatic SPTs often confound radiologists and referring clinicians with how to manage them.

Previously published papers have found that the incidence of asymptomatic SPTs is high [1, 14, 15]. In an extensive review of the English literature, 2744 cases of SPTs were reported, including 593 asymptomatic cases [2]. Interestingly, a high incidence of SPT has been observed among asymptomatic patients in our hospital. Herein, the imaging features and clinical characteristics of SPTs in asymptomatic patients are described and compared with those of symptomatic patients to help radiologists recognize the tumors and provide a more confident diagnosis.

## Methods

### Patient selection

Our institutional review board approved of this retrospective study, and the requirement for informed consent was waived. A total of 109 consecutive patients in our institution with pathologically confirmed SPTs who had undergone MDCT imaging in the immediate preoperative period (within 14 days before surgery) from October 2008 to October 2016 were retrospectively evaluated. Asymptomatic SPT was defined as an unexpected pancreatic tumor detected during clinical investigation of an unrelated condition and incidentally detected by one or more imaging methods or a screening program. Patients were divided into 2 groups: 49 were asymptomatic (mean age, 33.3 years; range, 11–64 years) and 60 were symptomatic patients (mean age, 31.0 years; range, 14–65 years). After each operation, patients were assessed clinically and then by ultrasonography and MDCT upon follow up.

### CT examination

All CT investigations were carried out by MDCT of the abdomen, and different MDCT machines were used over the 8-year period: 47 on 16-slice and 62 on 64-slice MDCT scanner (Lightspeed 16 or Lightspeed 64; GE Medical Systems, Milwaukee, WI, USA). After fasting for at least 4 h before scanning, all patients were administered 500–800 mL of water 30 min prior to imaging, and an additional 250–300 mL of water was given immediately prior to imaging to achieve adequate distension of the stomach and duodenum.

All patients were given nonionic iodinated contrast medium (Ultravist 300, Bayer Schering, Berlin, Germany) at a concentration of 300 mg iodine/mL administered at a flow rate of 3–4 mL/s through an 18-gauge intravenous catheter placed in the antecubital vein, followed by a 40 mL bolus of saline solution. The contrast material was delivered at a dose of 1.5–2 mL/kg body weight. Sixty-seven patients underwent triple-phase CT during the nonenhanced, arterial, pancreatic, and portal venous phases, while 42 patients underwent dual-phase CT during the nonenhanced, pancreatic, and portal venous phases. The Z-axis coverage of unenhanced and arterial (pancreatic) phase scans was from the domes of the diaphragm to the anterior superior iliac spines; the coverage of the portal venous phase scans was to the ischial tuberosities.

The scanning parameters for both noncontrast and contrast-enhanced CT examination were as follows: tube peak voltage, 120 kV; tube current, 250 mAs; gantry rotation time, 0.5 s; 1.0 pitch; 0.625–4 mm collimation; slice thickness 3.0–4.0 mm, slice interval, 2.5 mm. The delay times of the arterial, pancreatic, and portal venous phase were 30–35, 45, and 60–65 s, respectively, from the beginning of intravenous infusion. Reformed images (coronally and sagittally) were obtained using multiplanar reformation technique on the advanced workstation.

### Imaging analysis

MDCT images were retrospectively reviewed on the hospital picture archiving and communication system by two senior abdominal radiologists with 10 and 8 years of experience in abdominal CT. The reviewers were blinded to the clinical and pathological data of all of the pancreatic lesions but were aware that all patients had a presumptive diagnosis of SPT. Discrepancies between the readers were resolved by consensus after joint re-evaluation of the images. The examinations were reviewed in random order, with a time interval of at least 1 month and a mean interval of 21 d.

For qualitative analysis, all tumors were assessed for the following features: (1) tumor shape: oval/round or lobulated; (2) tumor location: head and neck, body, and tail of the pancreas; (3) calcifications: present or absent; (4) encapsulation: present or absent; (5) tumor composition: existence of solid and cystic components and fraction of the tumor cystic versus solid material (more than 50% solid or less than 50% solid); (6) attenuation on the pancreatic phase: internal density of the tumor was compared with that of the surrounding pancreas and described as hypo-, iso-, or hyperattenuation; (7) enhancement pattern during the pancreatic phase: enhancement pattern of the tumor was classified as peripheral and persistent or central and persistent during multi-phasic dynamic MDCT; (8) parenchymal atrophy; (9) dilatation of the main pancreatic duct: positive if the diameter of the main pancreatic duct exceeded 3 mm, negative otherwise. All measurements were repeated three times at three contiguous imaging levels, and average values were calculated to ensure consistency. In addition, patient age, sex, symptoms, and duration of symptoms were reviewed. Images were evaluated in terms of atrophy of the pancreas, pancreatic and bile duct dilatation, spread to regional vasculature, lymphadenopathy, adjacent organs, and distant metastasis.

For quantitative analysis, the following features were assessed: (1) tumor size: longest axial diameter in either the axial, coronal, or sagittal planes, depending on the spatial orientation of the tumor; (2) dilatation of the main pancreatic duct: positive if the diameter of the main pancreatic duct exceeded 3 mm.

### Surgical and pathologic analysis

Available records of clinical presentation, reason for detection, and surgical and final pathological diagnosis were identified from the hospital electronic medical records and reviewed for all cases. CT imaging features were correlated with gross pathologic and histologic findings in each case.

### Statistical analysis

Clinical features (sex, age, surgical procedure, surgical approach, and malignancy) and conventional MSCT features (tumor shape, tumor size, location, calcification, encapsulation, tumor composition, attenuation on pancreatic phase, enhancement pattern during the pancreatic phase, parenchymal atrophy, and dilatation of main pancreatic duct) were analyzed.

Quantitative variables were expressed as mean ± standard deviation. Categorical variables were expressed as counts, and statistical comparisons between the two groups were made using the χ2 and t-tests for continuous variables. A *P*-value of < 0.05 was considered to indicate statistically significant differences, and all calculations were performed using Statistical Package for the Social Sciences software (SPSS version 13.0; SPSS Inc., Chicago, IL, USA).

## Results

### Clinical features

This study included data from 49 asymptomatic and 60 symptomatic patients with a mean age of 30.0 years (range, 11–65 years). Fifteen patients were asymptomatic before 2012, while 34 patients, or > 2/3 of the asymptomatic group, were incidentally discovered between 2013 and 2016. The specific reasons for the radiographic evaluations of SPTs of the asymptomatic patients are given in Table 1. The three most frequent indications for imaging included routine health examination (18 patients, 36.7%), various screening purposes (12 patients, 24.5%), and traumatic injury (9 patients, 18.4%). The clinical characteristics of the 109 patients are summarized in Table 2. No statistically significant difference was observed in terms of clinical factors between SPTs in asymptomatic and symptomatic patients. Both sexes were similar in age, and few surgical procedures were specific. All 109 patients underwent different curative resections according to the preoperative diagnosis and intra-operative frozen section. No significant differences were found between asymptomatic and symptomatic patients with respect to surgical procedures, surgical approach, or malignant SPTs. Only eight cases (16.3%) underwent surgery with laparoscopy among symptomatic patients, and all of them received distal pancreatectomy. Fourteen cases (18.3%) were diagnosed as malignant SPTs in asymptomatic and symptomatic patients on account of histologic evidence of adjacent tissue invasion or metastasis to the spleen (*n* = 6), duodenum (*n* = 3), kidney (*n* = 1), vessel encasement (*n* = 3), and liver (*n* = 1).

**Table 1:** Most common initial presentations of asymptomatic SPTs

Presentation	Number	Percent
Health examination	18	36.7
Screening/surveillance	12	24.5
Trauma/emergency	9	18.4
Postoperative/follow-up	6	12.2
Others	4	8.2
Total	49	100

**Table 2:** Comparison of clinical characteristics of asymptomatic and symptomatic SPTs

Variables	Asymptomatic (*n* = 49)	Symptomatic (*n* = 60)	*P*-value
Age (years)	33.3 ± 12.4	31.0 ± 13.9	0.357
Sex (Male/Female)	10/39	9/51	0.613
Surgical procedure, n			0.983
Whipple’s procedure or PPPD	13	17	
DP + SPL	16	21	
DP only	9	11	
Enucleation	4	5	
SP	7	6	
Surgical approach, n			0.806
Laparoscope	8	11	
Open	41	49	
Malignant, n	6	8	0.866

*SD* indicates standard deviation; *PPPD* pancreaticoduodenectomy, *DP* distal pancreatectomy, *SPL* splenectomy, *SP* segmental pancreatectomy

Follow-up data were obtained from outpatient records and telephone interviews. The follow-up period ranged from 4 months to 97 months (median follow-up, 62 months), and all patients were alive at the end of this period with no evidence of disease recurrence or distant metastasis.

### Imaging features

The CT features of SPTs observed in asymptomatic (Fig. 1) and symptomatic (Fig. 2) patients are summarized in Table 3. Except for tumor size, the imaging features of SPTs in asymptomatic and symptomatic patients did not show significant differences in terms of tumor shape, location, calcification, encapsulation, tumor composition, attenuation on the pancreatic phase, enhancement pattern during the pancreatic phase, parenchymal atrophy, and dilatation of the main pancreatic duct. The mean diameters of tumors in asymptomatic and symptomatic patients were 5.8 cm (range, 1.0–11.0 cm) and 7.4 cm (range, 2.5–17.0 cm), respectively, and the mean tumor size in symptomatic patients was significantly larger than that in asymptomatic patients (7.4 cm vs. 5.8 cm; t = 2.303, *P* = 0.023). No predominant location or shape of the SPTs was found in asymptomatic patients, and 20 (20/49) patients of this group showed complete and smooth encapsulation on images; the other 29 asymptomatic SPTs showed focal discontinuity or invisible capsule on both unenhanced and enhanced images. Calcification was detected in 10 asymptomatic patients (10/49; 20.4%), specifically at the periphery (*n* = 5), center (*n* = 3), and capsule (*n* = 2) of the tumors. On MDCT, the tumors of asymptomatic and symptomatic patients could be divided into three types according to density, namely, cystic, solid, and solid–cystic component (mixed). Multi-phasic dynamic MDCT analysis was thus performed. Compared with the CT attenuation characteristics of the pancreatic parenchyma, pancreatic phase images showed tumors with hyperattenuation (*n* = 7), isoattenuation (*n* = 13), and hypoattenuation (*n* = 29) in asymptomatic patients; 17 cases (17/49) in this group manifested peripheral enhancement with progressive fill-in while the remaining 32 cases (32/49) showed central and progressive fill-in of the pancreas during the pancreatic phase after contrast material administration.

**Fig. 1:** Abdominal CT scans of asymptomatic SPT in a 31-year-old woman. **a** Unenhanced CT scan showing a 9.0 cm oval mass at the head of the pancreas with homogeneous isoattenuation. Calcification is seen at the periphery of the mass. **b** Scan obtained during the pancreatic phase. **c** Scan obtained during the hepatic venous phase showing a mass with a progressive fill-in enhanced pattern. **d** Coronal pancreatic phase CT image showing complete, smooth, and delayed enhancement of the tumor pseudocapsule

**Fig. 2:** Abdominal CT scans of symptomatic SPT in a 21-year-old woman. **a** Unenhanced CT scan showing a large heterogeneous mass in the body of the pancreas, dilatation of the pancreatic duct and parenchymal atrophy (arrow) distal to the mass lesion in the body of the pancreas. **b** Scan obtained during the pancreatic phase. **c** Scan obtained during the hepatic venous phase showing mostly solid and small cystic areas at the center and a cystic mass without significant contrast enhancement. **d** Coronal pancreatic phase CT image showing dilatation of the pancreatic duct and parenchymal atrophy (arrow) distal to the mass lesion in the body of the pancreas

**Table 3:** Imaging characteristics of asymptomatic and symptomatic SPTs

Variables	Asymptomatic (*n* = 49)	Symptomatic (*n* = 60)	*P*-value
Shape, n			0.337
Oval or round	21	32	
Lobulated	28	28	
Size (cm)	5.8 ± 3.4	7.4 ± 3.5	0.023
Tumor location, n			0.847
Head, and /or neck	27	31	
Body, and /or tail	22	29	
Calcification, n			0.818
Present	10	14	
Absent	39	46	
Encapsulation, n			0.701
Present	20	27	
Absent	29	33	
Tumor composition, n			0.564
More than 50% solid	22	31	
Less than 50% solid	27	29	
Attenuation on pancreatic phase, n			0.697
Hyperattenuation	7	11	
Isoattenuation	13	19	
Hypoattenuation	29	30	
Enhancement pattern during pancreatic phase, n			0.328
Peripheral and persistent enhancement	17	27	
Central and persistent enhancement	32	33	
Parenchymal atrophy, n			0.741
Present	4	6	
Absent	45	54	
Pancreatic duct dilatation, n			0.616
Present	5	8	
Absent	44	52	

*SD* indicates standard deviation

Although no marked difference in terms of prevalence of parenchymal atrophy or pancreatic ductal dilatation was observed between the two groups, all SPTs showed low prevalence of associated parenchymal atrophy (9%) and pancreatic duct dilatation (11.9%).

## Discussion

Although an increasing number of studies concerning SPTs of the pancreas have been published, little information is available on the clinical and MDCT manifestations of SPTs in asymptomatic and symptomatic patients due to their rarity. This study suggests that SPTs in asymptomatic patients are gradually being identified with greater frequency given current innovations in diagnostic imaging. To the best of our knowledge, the current research is the largest single-center study to analyze the imaging features and clinical characteristics of SPTs in asymptomatic patients to date. Furthermore, no prior report comparing the imaging features of asymptomatic and symptomatic patients has yet been published. This study reveals that, except for tumor size and management of clinical factors, the radiological features of SPTs in asymptomatic and symptomatic patients are similar. The diagnosis of SPT in asymptomatic patients is a relatively recent clinical phenomenon. However, many surgeons are still unfamiliar with asymptomatic SPT and its unique imaging characteristics, which can lead to challenges in diagnosis and treatment. Correct diagnosis of SPT is of utmost importance since the tumor has low malignancy potential, and, with the appropriate treatment, patients could have a long life expectancy.

SPT currently constitutes about 2–3% of all primary pancreatic tumors. Due to advanced imaging technologies and increasing awareness of this tumor, the number of SPTs reported in the literature has seen a sevenfold increase since 2000, with 90% of the incidental cases detected within the last 12 years [2]. With time, asymptomatic SPTs are increasing likely to be discovered. Xu et al. previously reported that the proportion of asymptomatic SPTs is as high as 71.1% [15]. In our retrospective series, 49 (49/109, 45%) of the asymptomatic SPTs were eventually discovered (34 patients, > 2/3 incidentally discovered from 2013 to 2016). The exact incidence of SPT in asymptomatic patients is not known.

SPTs in asymptomatic patients are often initially discovered during clinical evaluations of a wide variety of symptoms. In the present series, a diagnosis of SPT was often made after imaging for physical examination, traumatic injury, and various screening purposes, all of which are in agreement with the series of Law et al. [2].

SPTs, including asymptomatic ones, can occur in every part of the pancreas (body/tail, 49%; head/neck, 55%). No predominant location of SPTs was indicated for asymptomatic patients, and the locations of SPTs showed no remarkable difference between the two groups in the present study. The tumor size of SPTs in symptomatic patients were inclined to be larger than those in asymptomatic patients (7.4 cm vs. 5.8 cm; *P* = 0.023), which supports the rationale behind the widespread use of multislice CT scanning.

The imaging characteristics of SPTs include a large size, mass with mixed solid and cystic components, encapsulated appearance, presence of hemorrhage, and peripheral contrast enhancement corresponding to a fibrous pseudocapsule [2, 16–20]. In our series, except for tumor size, the imaging features of SPTs in asymptomatic and symptomatic patients showed no significant differences. The typical radiological features of SPTs in asymptomatic patients include a large, well-circumscribed tumor, solid and cystic components, (often) fibrous pseudocapsules, and peripheral contrast enhancement. Recognition of the radiological features of SPT in asymptomatic patients compared with those of typical SPT in symptomatic patients should assist in correct differentiation of SPT from other pancreatic tumors. Familiarity with the characteristic CT appearances and clinical characteristics of SPTs in asymptomatic patients will help radiologists provide more accurate diagnoses with better confidence. However, typical radiological findings can also be an indication for surgery [6].

In a 2010 WHO report, SPTs were classified as a potential malignant tumors. Most reported cases of SPTs are known to be benign; however, malignancy does occur in 9–15% of the cases discovered [6]. Previous studies have suggested that some clinicopathological parameters found male patients, such as large tumor size and Ki-67 expression, are indicators of tumor aggressiveness and poor prognosis [14, 21, 22]. Some researchers have also reported that the malignancy potential of SPTs cannot be predicted before surgery by age, sex, tumor size, or tumor markers [13]. To date, little consensus has been reached in predicting the malignant behavior of SPTs. In addition, no consensus regarding the clinical risk factors for recurrence has yet been established [15].

Surgery is the main therapeutic modality for low-grade malignant SPTs. Once SPT is diagnosed in asymptomatic patients, given the excellent prognosis and low-grade malignancy potential of the tumor, less-aggressive surgical resection of the primary lesion is proposed [2, 6, 9, 10]. Surgery with sparing of as much pancreatic tissue as possible is the optimal treatment and offers an excellent prognosis, even in the presence of distant metastases or local invasive effects. A good prognosis is expected after surgical resection of primary tumors; even patients who exhibit distant metastasis have good prognoses as long as the metastatic lesions are resected completely. However, pancreas- or spleen-preserving procedures may be considered in experienced centers [13]. In our hospital, the surgical management of SPTs performed in asymptomatic patients is similar to that in symptomatic patients. Guidelines for the surgical treatment of SPT remain a challenging field that requires further research. All asymptomatic and symptomatic patients with SPTs remained alive with no evidence of disease recurrence at the end of follow up.

The current study presents some limitations. First, our study is retrospective in nature and may include selection bias. Thus, other studies, such as a prospective multi-center studies including a sufficient number of patients with long-term follow up, are needed to validate our result. Second, the rarity of SPTs in asymptomatic patients results in limited experience in individual institutions. The number of patients included in this work is inadequate to draw definitive conclusions. Larger case series and further studies are needed to support our conclusions. Third, because the cases were collected over 8 years, different types of MDCT scanners and different CT parameters were employed. However, as the procedures for reconstruction of section thickness were similar, we believe that the imaging features studied should not significantly differ.

## Conclusions

In summary, the data presented in this study demonstrate that an increasing number of patients are being identified with asymptomatic SPTs of the pancreas. The current research is the largest single-center study to demonstrate SPTs in asymptomatic patients. Compared with those in symptomatic patients, tumors in asymptomatic patients are smaller in size. Both asymptomatic and symptomatic patients showed the same radiological features. Asymptomatic patients with typical imaging prominently showed enhancement patterns typical of SPTs, such as heterogeneity within a well-circumscribed tumor with a fibrous pseudocapsule. In combination with clinical findings, the typical radiological features of SPT in asymptomatic patients may help radiologists provide correct diagnoses and differentiate the tumor from other pancreatic neoplasms. Once diagnosed, given the excellent prognosis and low-grade malignancy potential of SPTs, less-aggressive surgical resection of the primary lesion is proposed. Multicenter cooperation is necessary to confirm our conclusions.

## Abbreviations

DP: Distal pancreatectomy
MDCT: Multi-detector computed tomography
MRI: Magnetic resonance imaging
PPPD: Pancreaticoduodenectomy
SD: Standard deviation
SP: Segmental pancreatectomy
SPL: Splenectomy
SPT: Solid pseudopapillary tumor
